RETRACTED

# The Efficacy of Mannitol Combined with 6-Aminocaproic Acid in the Treatment of Patients with Cerebral Hemorrhage and Its Impact on Immune Function

**DOI:** 10.1155/2022/7396310

**Published:** 2022-07-12

**Authors:** Buxian Tian, Bohan Tian, Yuhong Zhang

**Affiliations:** ^1^Department of Neurology, First Affiliated Hospital of Jinzhou Medical University, Jinzhou 121001, Liaoning, China; ^2^Class 2017 imaging department, Jinzhou Medical University, Jinzhou 121001, Liaoning, China; ^3^Department of Neurology, Jinzhou General Hospital, Jinzhou, Liaoning, China

## Abstract

**Objective:**

To determine the efficacy of Mannitol combined with 6-aminocaproic acid in the treatment of patients with cerebral hemorrhage, as well as its impact on the immune system.

**Methods:**

The study subjects consisted of 122 patients with early intracerebral hemorrhage treated in our hospital from April 2019 to April 2022. Based on the different admission times, the participants were randomly divided into the control group and the study group in a ratio of 1:1. 6-Aminocaproic acid was used to treat patients in the control group, while Mannitol along with 6-aminocaproic acid was used to treat patients in the study group. Short form-36 health survey (SF-36) scores, hematoma volume changes, National Institutes of Health Stroke Scale (NIHSS), and Mini-Mental State Examination (MMSE) scores, clinical efficacy, and changes in the immune function in patients from the two groups were analyzed and compared.

**Results:**

The total efficacy of treatment in the study group was significantly higher than that in the control group (*x*^2^ = 9,375, *P* < 0.001). Patients in the study group had significantly higher scores in social function, mental health, physical function, and physiological function compared to those in the control group (*P* < 0.05). After treatment, there was a significant reduction in NIHSS scores in patients from both groups, but a greater reduction was seen in patients from the study group (*P* < 0.05). After 2 weeks of treatment, the volume of cerebral edema was significantly smaller in patients from the study group than in those from the control group (*P* < 0.05). Before treatment, there was no significant difference in the number of CD4+ and CD8+ T lymphocytes between patients in the two groups. However, after treatment, patients in the study group had higher numbers of CD4+ T lymphocytes and lower numbers of CD8+ T lymphocytes compared to those in the control group (*P* < 0.05).

**Conclusions:**

The combination of Mannitol and 6-aminocaproic acid appears to be very efficacious in the treatment of cerebral hemorrhage. It improves immune function, reduces neurological damage, and minimizes the volume of cerebral edema.

RETRACTED

## 1. Introduction

Clinically, hemorrhage associated with nontraumatic brain injury that is caused by rupture of blood vessels in the brain is referred to as cerebral hemorrhage. It is a chronic cerebrovascular disorder [1, 2] that is very common in the field of neurology. It accounts for about 30% of all strokes [3], and causes significant morbidity and mortality. It usually occurs in middle-aged or elderly patients with poorly controlled hypertension and is associated with a lot of complications. It poses a serious threat to the health of patients [4, 5]. Hemorrhage is frequently accompanied by somatic dysfunction due necrosis of neurons [6]. The clinical symptoms and their severity depend on which arterial territory is involved and the size of the lesion [7]. The typical presentation occurs over minutes, affects an identifiable area of the brain and is “negative” in character (i.e., abrupt loss of function without positive features such as abnormal movement). Provided there is a clear history of this, the chance of a brain lesion being anything other than vascular is 5% or less. Some patients may also experience sequelae such as language, cognitive, and motor impairments. Symptoms are sudden in onset and if the treatment is delayed, the mortality rate can be very high. Therefore, an effective treatment plan is crucial to the patient's survival. If not devised in time, death could result [8].

Currently, treatment of cerebrovascular diseases is primarily pharmacological. 6-aminocaproic acid, an inhibitor of fibrinolysis, is the most commonly used hemostatic drug in the treatment of cerebral hemorrhage [9]. However, using this drug alone cannot reduce intracranial blood pressure fast enough, leading to only a small improvement in the patient's condition. Consequently, the concomitant use of antihypertensive agents when treating such patients is critical. To understand the mechanism of action of 6-aminocaproic acid, one must have a basic understanding of the physiology of coagulation. The main component of a hemostatic plug is fibrin. Fibrin can be degraded by plasmin, which is the active form of plasminogen. The conversion of plasminogen to plasmin relies on the action of plasminogen activators. 6-aminocaproic acid works mainly by inhibiting plasminogen activators, thus preventing the conversion of plasminogen to its active form, plasmin. By doing so, the drug inhibits dissolution of fibrin, thus, maintaining the hemostatic plug [10]. Rapid injections of large volumes of Mannitol intravenously may cause a buildup of Mannitol in the body. This leads to a rapid increase in the blood volume, resulting in heart failure, dilutional hyponatremia and even hyperkalemia. Excessive diuresis can also lead to hypovolemia, which aggravates oliguria [11]. Mannitol is an isomer of sorbitol that acts as an osmotic diuretic, resulting in a rapid reduction of intracranial pressure. It also induces dehydration [12]. In recent years, compression medicine has been used to treat and control cerebrovascular diseases. Currently, there are few studies on the efficacy of Mannitol and 6-aminocaproic acid in the treatment of cerebral hemorrhage. It is against this backdrop that our study aims to determine the clinical efficacy of Mannitol and 6-aminocaproic acid in the treatment of intracerebral hemorrhage, with a view to providing a reliable reference for future clinical application.

RETRACTED

## 2. General Information and Methods

### 2.1. General Information

The study included 122 patients with early cerebral hemorrhage who were admitted to our hospital from April 2019 to April 2022. The patients were randomly assigned to either the control or the study group based on the time of admission. There were 61 patients in each group. All patients were informed of this study, and all of them provided informed consent. The study was reviewed and approved by the Medical Ethics Committee of the First Affiliated Hospital of Jinzhou Medical University before it began (Approval No. 20196104).

#### 2.1.1. Inclusion Criteria

Patients who met the following criteria were included in this study:

1. Patients who had intracerebral hemorrhage that met the criteria set forth in the *Standards of the 4th National Academic Conference on Cerebrovascular Diseases* [13].
2. Patients who did not suffer from other serious illnesses.
3. Patients who were never transferred to other hospitals for the entirety of this study, and whose information was complete.
4. Patients who saw a doctor within 24 hours of symptom onset.

#### 2.1.2. Exclusion Criteria

The following patients were excluded from the study:

1. Patients with severe liver and kidney dysfunction.
2. Patients who were allergic to either 6-aminocaproic acid or amnnitol.

### 2.2. Methods

All patients were given routine treatment following diagnosis: monitoring and regulating blood pressure, maintaining stillness, maintaining smooth breathing, maintaining the balance of various trace elements in the body, nutritional support, use of antihypertensive agents, hemostasis, and other symptomatic treatments. Patients in the control group received continuous intravenous infusions of 6-aminocaproic acid at a dosage of 24 g/d during the first week of treatment, followed by gradual reductions to 8 g/d thereafter. In the event of a sudden drop in the blood pressure or cardiac arrest, the drug should immediately be discontinued and emergency treatment must be administered. Patients in the study group were treated in much the same way as those in the control group, but Mannitol was also added to the treatment regimen. Mannitol was administered twice a day by an intravenous drip in a dosage of 5 ml. The time of each drip was controlled to about 30 minutes. The patient's intracranial pressure was measured regularly, and if it fell to below 20 mmHg, the drug was discontinued.

RETRACTED

All patients were observed for 2 weeks.

### 2.3. Observational Indicators

1. *Comparison of Clinical Efficacy between the Two Groups*. Markedly effective: patients report complete disappearance or significant improvement in symptoms, and they do not exhibit any disability. Effective: Patients report significant improvement in symptoms, with mild disability. Ineffective: Patients report no improvement or worsening of symptoms, with severe disability. Total efficacy rate = (markedly effective + effective) number of cases/total number of cases × 100%.
2. Quality-of-life score: the quality-of-life score (SF-36) primarily focused on four dimensions, each worth 100 points [14]. The higher the patient's score, the better their quality of life.
3. Neurological function: the NIHSS was used to assess neurological damage. The higher the score, the more severe the damage [15]. We assessed the patient's cognitive function using the MMSE, which has a total score of 30. The lower the score, the worse the patient's cognitive function [16].
4. Cerebral edema volume: CT scans of the patient's head were obtained before initiation of treatment and after 2 weeks after treatment, and calculated the volume of cerebral edema using the Tada formula.
5. Immune function: flow cytometry was used to measure the number of CD4+ and CD8+ T lymphocytes.

### 2.4. Statistical Analysis

SPSS 24.0 was used as the data analysis software. Measurement data was expressed as $\left(\bar{x}\pm s\right)$, and the independent *t*-test samples were used. Enumeration data was expressed as the number of cases (%), and the chi-square test was used. Statistical significance was assumed at a *P* value <0.05.

## 3. Results

### 3.1. Comparison of the General Information

There was a total of 37 males and 24 females in the control group, aged between 41 and 82 years, with an average of 61.08 ± 5.44 years. This group had 34 cases of putamen hemorrhage and 27 cases of lobar hemorrhage. There was a total of 35 males and 26 females in the study group, aged between 40 and 82 years, with an average age of 60.37 ± 5.49 years. This group had 35 cases of putamen hemorrhage and 28 cases of lobar hemorrhage. There was no significant difference in the general data of patients from the two groups (*P* > 0.05).

RETRACTED

### 3.2. Comparison of Clinical Efficacy

The total clinical efficacy rate was 95.08% in the study group and 78.69% in the control group. Compared to the control group, the study group had a significantly higher finite rate (**X**^2^=9.735, *P* < 0.001). See Table 1 for more details.

### 3.3. Comparison of Quality-of-Life Scores

Patients in the study group scored significantly higher in social function, mental health, physical function, and physiological function compared to those in the control group after treatment (*P* < 0.05). See Table 2 for details.

### 3.4. Comparison of Neurological Function

There was a reduction in the NIHSS score of patients from both groups following treatment. However, a greater decrease was seen in the study group than in the control group (*P* < 0.05). There was also no significant difference in the MMSE score of patients from the two groups before treatment. After treatment, there was an increase in the MMSE score in patients from both groups, but a greater increase was seen in the study group than in the control group (*P* < 0.05). See Table 3 for details.

### 3.5. Comparison of Changes in the Cerebral Edema Volume

The volumes of cerebral edema in the two groups of patients after 2 weeks of treatment were significantly smaller than those before treatment. Patients in the study group had significantly smaller volumes than those in the control group (*P* < 0.05). See Table 4 for details.

### 3.6. Comparison of Immune Function

Before treatment, there was no significant difference in the numbers of CD4^+^ and CD8^+^ T lymphocytes between the two groups of patients. Following treatment, patients in the study group had higher numbers of CD4^+^ T lymphocytes and lower numbers of CD8^+^ T lymphocytes compared to those in the control group (*P* < 0.05). See Table 5 for details.

## 4. Discussion

Intracerebral hemorrhage usually occurs when there is a sudden rise in the blood pressure that ruptures an artery and causes bleeding. There are many other types of cerebral hemorrhage, which can be caused by numerous factors [17, 18]. Patients usually have no prodromal symptoms, but a few may have dizziness, headache, and weakness of the limbs. The symptoms reach their peak within minutes or hours of onset. As earlier alluded to, the nature of symptoms as well as their severity depends on the artery involved [19]. Failure to provide quick interventions can endanger the patient's life [20]. Treatment of cerebral hemorrhage can be medical or surgical, usually the former, unless the condition is critical or if a secondary cause is found and there are indications for surgery [21]. Medical management mainly focuses on controlling bleeding and reducing intracranial pressure. If the patient is currently taking anticoagulants (e.g., warfarin) or antiplatelets (e.g., clopidogrel), then the patient may be given other drugs or blood transfusions to counteract the effects of the anticoagulants or antiplatelets. The patients may also be given drugs to lower systemic and intracranial blood pressure, prevent vasospasm or prevent seizures [22, 23]. Once the bleeding in the brain has stopped, treatment usually involves supportive medical care while the hematoma gets absorbed [24]. If the bleeding is extensive, the surgeon may perform surgery to remove the hematoma and relieve the pressure it exerts on the brain [25]. In patients with cerebral hemorrhage, hemostatic drugs should be administered quickly. 6-aminocaproic acid is an antifibrinolytic drug [26], and studies have shown that antifibrinolytic drugs can reduce bleeding by more than 50% [21, 27, 28]. Upon intravenous administration, this medication acts directly on the site of the lesion. Researchers have shown that when Mannitol is used as a supplementary therapy in patients with cerebral hemorrhage, the clinical outcome is greatly improved. Mannitol is commonly used as an osmotic diuretic in the clinical setting. It works by enhancing the kidneys' ability to eliminate water from the body, thus reducing blood volume and ultimately, intracranial pressure [29].

RETRACTED

The results of this study have shown that there were no statistically significant differences in neurological function score or cognitive function score between patients from the two groups prior to the treatment. There was a reduction in the NIHSS score of patients from both groups following the treatment, but a greater decrease was seen in the study group than in the control group. There was also an increase in the MMSE score in patients from both groups following treatment, but a greater increase was seen in the study group than in the control group. Following the treatment, the quality-of-life scores of patients in the study group were higher than those of patients in the control group. Researchers found that combining the two drugs reduced the severity of damage to neurons and improved the cognitive function. This in turn improved the patient's quality of life and the prognosis. Other studies have also arrived at a similar conclusion [21]. In addition to symptoms secondary to hemorrhage, the immune system also plays an important role. In order to assess changes in the immune function of patients, CD4^+^ and CD8^+^ expression levels were evaluated. Our results show that there was no significant difference in the numbers of CD4^+^ and CD8^+^ T lymphocytes between patients in the two groups before the treatment. Following the treatment, patients in the study group had higher numbers of CD4^+^ T lymphocytes and lower numbers of CD8+ T lymphocytes compared to those in the control group. This indicates that combining the two drugs can greatly improve the patient's immune function. It is sometimes possible to determine the severity of acute cerebral hemorrhage from the volume of cerebral edema. We measured the volume of cerebral edema after 2 weeks of treatment, and found that patients in the study group had small volumes than those in the control group. The total clinical efficacy rate was 95.08% in the study group and 78.69% in the control group. A significantly higher finite rate was observed in the study group compared to the control group.

RETRACTED

It can, therefore, be concluded that Mannitol can improve clinical outcomes and reduce cerebral edema in patients with intracerebral hemorrhage. This finding is the same as what is reported in the hypothesis [30]. The reason for this may be that patients with mild hemorrhages have a small amount of bleeding, and 6-aminocaproic acid is used to stop the bleeding as quickly as possible, thus reducing the possibility of subsequent bleeding and improving the clinical outcomes. On the other hand, patients with severe diseases have a larger amount of bleeding and significantly higher intracranial pressure than those with mild hemorrhages. Currently, Mannitol is used as a supplement to 6-aminocaproic acid, and evidence suggests that it increases the clinical efficacy of treatment and prevents further deterioration [31–33]. The reason for this may be that Mannitol is able to facilitate the flow of cerebrospinal fluid and water in the brain tissue into the circulation, thus reducing cerebral oedema and lowering intracranial pressure. It also improves cerebral blood circulation, reduces the number of inflammatory mediators in the brain tissue, and increases mean arterial pressure, hence improving neurological function.

Patients with cerebral hemorrhage can be treated with Chinese medicine, including herbal medicine, acupuncture, massage, and a combination of Chinese and western medicine [34]. Chinese medicine emphasizes syndrome differentiation and treatment. If there are symptoms of hyperactivity of the liver yang such as irritability, red eyes, and a stringy pulse, Tianma Gouteng decoction can be used to calm the liver and relieve wind. If there is wind-phlegm or phlegm-heat manifestations such as coughing white phlegm or sticky phlegm, Ditan Tongluo decoction can be used to expel phlegm and activate collaterals. If patients have symptoms of Qi (breath power) deficiency and blood stasis such as laziness, fatigue, red tongue, and a stringy pulse, Buyang Huanwu decoction can be used to nourish Qi and activate the blood. Also, one can take Qi and blood drugs on weekdays to improve one's constitution [35–37]. In addition to oral herbal tonics, acupuncture can also be used to invigorate the blood and eliminate blood stasis, and to benefit and tonify the Qi [38].

RETRACTED

The relatively small sample size of our study may make the results regionally heterogeneous, with a high probability of error. Secondly, recovery following cerebral hemorrhage is a long process, and our study lacks long-term follow-up to determine the prognosis. In future studies, we hope to conduct an in-depth analysis of the molecular mechanisms and signaling pathways that are responsible for the results.

## 5. Conclusion

The combination of Mannitol and 6-aminocaproic acid appears to be very efficacious in the treatment of cerebral hemorrhage. It improves immune function, reduces neurological damage, and minimizes the volume of the cerebral edema. This treatment regimen is one that definitely deserves more widespread promotion and clinical application.

## Figures and Tables

**Table 1:** Comparison of efficacy of treatment between the two groups [*n*(%)]_._

Group	*n*	Effective	Ineffective	Total efficacy rate
Control group	61	32	13	48 (78.69%)
Study group	61	31	3	58 (95.08%)
*X* ^2^				9.735
*P*				<0.001

**Table 2:** Comparison of quality-of-life scores between the two groups after treatment [$\left(\bar{x}\pm s\right)$, points].

Group	*n*	Social function	Mental health	Physical function	Physiological function
Control group	61	76.31 ± 4.15	81.39 ± 4.27	80.71 ± 4.53	83.26 ± 3.62
Study group	61	93.25 ± 6.24	92.74 ± 4.90	92.77 ± 5.18	93.52 ± 5.71
*t*		18.491	10.629	12.537	11.352
*P*		<0.001	<0.001	<0.001	<0.001

**Table 3:** Comparison of neurological impairment in the two groups [$\left(\bar{x}\pm s\right)$, points)].

Group	*n*	NIHSS score		MMSE score	
		Before treatment	After treatment	Before treatment	After treatment
Control group	61	23.48 ± 3.07	15.65 ± 2.91	21.13 ± 1.65	24.21 ± 1.84
Study group	61	23.44 ± 3.11	10.37 ± 2.30	21.09 ± 1.49	27.63 ± 2.37
*t*		0.067	6.337	0.086	3.693
*P*		0.985	0.021	0.947	0.013

**Table 4:** Comparison of changes in the cerebral edema volume between the two groups [$\left(\bar{x}\pm s\right)$, cm^2^].

Group	*n*	Before treatment	Two weeks after treatment
Control group	61	25.36 ± 3.81	19.37 ± 2.63
Study group	61	25.37 ± 3.85	14.31 ± 2.18
*t*		0.034	5.414
*P*		0.931	0.02

**Table 5:** Comparison of immune function between the two groups [$\left(\bar{x}\pm s\right)$, %].

Group	*n*	CD4^+^		CD8^+^	
		Before treatment	After treatment	Before treatment	After treatment
Control group	61	26.57 ± 3.37	30.32 ± 3.52	35.62 ± 3.84	30.64 ± 3.38
Study group	61	26.48 ± 3.29	34.77 ± 3.87	35.67 ± 3.91	27.85 ± 3.23
*t*		0.097	4.982	0.057	7.664
*P*		0.928	0.035	0.894	<0.001

RETRACTED

## Data Availability

All data generated or analyzed during this study are included in this published article.
